The article "Community Environmental Detection and Community Outdoor Space Health Promotion Based on Cloud Resource Scheduling Mechanism" was published in 2022. Journal: J Healthc Eng.

# Community Environmental Detection and Community Outdoor Space Health Promotion Based on Cloud Resource Scheduling Mechanism

**DOI:** 10.1155/2022/4454447

**Published:** 2022-01-04

**Authors:** Chunyu Pang, Zhen Guan

**Affiliations:** Northeast Forestry University, Harbin 150040, China

## Abstract

In the context of rapid economic growth, people's living standards are improving day by day, and China's urbanization process is also gradually accelerating. Urban renewal is a very complex project. The renewal and expansion of most cities in the country usually involve demolishing and rebuilding. This way of urban renewal only pays attention to the renewal efficiency of cities and towns, and ignores the health needs of residents, which will make community residents lack a sense of security, pleasure, comfort, and belonging to the community, and greatly reduce the quality of life and physical fitness of community residents. Building a healthy city is an important goal of today's society, and community is the basic unit of a city, so it is urgent to build a health-promoting community. We should pay attention to and study the social environment, the external space environment of residential areas, and the interaction between them, so as to make develop them in a healthy direction and create a healthy and positive community. Therefore, it is an urgent task to improve the community residents' attention to the above problems and build community outdoor space, which has very important practical significance. In this paper, we use the cloud resource scheduling mechanism and the Internet of things to study the healthy role of community outdoor space planning. Through the transplantation of embedded Linux system, the development of communication interface and the external acquisition sensing device, we collect the information of working status and running status, and transmit it to the database built in the cloud through the 4G module on the motherboard. Then, HTML + java script + CSS + JSON + Ajax technology is used to write the display interface and logical relationship, so that the data can be displayed on the mobile terminal and PC, which can provide a useful technical exploration for outdoor space planning. The community Internet of Things technology realizes the intelligent community environment detection, and the community cloud resource scheduling mechanism combined with the community Internet of Things can obtain the residents' help information in time and allocate the community outdoor resources in real time, which can not only meet the health needs of community members but also be conducive to the sustainable development of a health-promoting community. In addition, the cloud resource scheduling mechanism and the Internet of things also provide new ideas for the study of the health promotion research of community outdoor space planning.

## 1. Introduction

Community outdoor space is essentially a space defined differently from interior space. It refers to the open space between architectural groups in the community, including the neighborhood space outside the house, such as roads, sidewalks, covered elevators, stairs and passageways, the rest place attached to the residence, etc. Community space has a certain purpose and communication, which serves the public for the purpose of communication, viewing, leisure, and so on. The elements that constitute community outdoor space can be divided into two categories: one is the community residents living in the community; the other is to serve the physical environment of community residents, that is, the hard environment. The elements of hard environment include natural elements and space elements. The natural elements are mainly flowers and trees, and the space elements are mainly residential, public service facilities, road paving, sketch sculpture, activity, places, and so on. Community outdoor space serves community members, and the design should reflect the specific theme of the community. It should not only pay attention to the relevance of space but also meet the basic living needs of community residents [1–3]. With the development of times, people gradually begin to pursue a healthy life and pay more attention to the quality of the living environment. Therefore, whether the community outdoor space can meet the health needs of community residents has become one of the criteria for community quality assessment. Yin Pingping analyzed the outdoor space design of a commercial and residential project in Nanjing, and emphasized that livable design should fully respect the opinions of residents. Fangyuan conducted research on the problem of upgrading and transforming outdoor communication spaces in old communities, and put forward the idea of attaching importance to semipublic outdoor spaces, providing a new idea for the transformation of old communities. Wang Yuyan believes that the current design of the community outdoor space has the same drawbacks and put forward a series of design schemes from an aesthetic point of view, which enriched the design system in this field.

The health needs of community residents are reflected in three levels of psychology, physiology, and behavior. However, community outdoor space planning often fails to take into account the health needs of residents at different levels, which eventually forms a vicious circle, leading to the deterioration of community health and negative impact on the physical health of community residents [4–6]. On July 1, 1998, China's housing welfare system was abolished, and the housing reform that had lasted for more than ten years has entered the stage of housing construction market and currency privatization. At the same time, some Chinese real estate development companies are overly keen to profit from real estate, resulting in high-density building volume [7]. In some community squares, the green area is too small, and the high-density buildings result in poor natural lighting conditions [8]. Living in such an environment for a long time will cause stress, depression, and physical and mental health problems among the residents [9]. The resultant negative impact will destroy the quality of the entire living environment [10]. Nowadays, many new residential areas do not create favorable conditions for social interaction, nor do they effectively manage related community exchanges and other issues, resulting in a significant reduction in communication among residents, which makes it more difficult to ensure mutual help between neighbors in the traditional sense [11]. Mutual assistance and mutual love is sadly missing. To a certain extent, this environment of lack of communication will exacerbate the indifference in interpersonal relationships. At the same time, this will even increase the probability of residents suffering from mental illness, such as feeling lonely, depressed, and anxious [12]. If we do not pay attention to the abovementioned problems, it will inevitably bring about very serious consequences [13]. In recent years, there have often been news reports of elderly people living alone, dying alone at home, and depressed teenagers committing suicide at home. These tragedies are inseparable from the lack of a supportive social environment, and the depressive environment will make people lose their sense of belonging to the community [14].

Therefore, in order to improve the quality of life of residents, it is necessary to build a healthy community conducive to neighborhood communication, safety, pleasure, and comfort. Residents, as the main body of outdoor space service in the community, are connected with the social environment, resulting in communication between individuals, between individuals and groups, and between groups. Moreover, the community material space has a direct emotional connection with the community culture, regulating and managing the community material environment. Therefore, community planning should adjust the sequence composition of various living spaces in the community space environment according to different types of health needs, so as to give community members a health-promoting outdoor space environment. Community outdoor space can lead the community to form a spiritual connotation with characteristics, so that the material space has social attributes, thus forming a unique culture and values, and jointly constituting the outdoor space environment to promote health. In order to allow the healthy development of the community environment, this article will use the cloud resource scheduling mechanism and the Internet of Things to explore the healthy role of community outdoor space planning [15].

## 2. Cloud Resource Scheduling Mechanism and Internet of Things Technology

In this article, the use of cloud resource scheduling mechanism and the Internet of Things technology provides suitable spaces and places with certain facilities and environments for the behaviorists, makes the layout of outdoor facilities in the community more reasonable, monitors the exercise intensity of community residents in real time, and promotes the healthy development of the community, so that community residents can also have a sense of belonging, regional affiliation, and security in the external space of the community [16].

### 2.1. Community Cloud Resource Scheduling Mechanism

Cloud resource scheduling refers to the process of adjusting resources among different resource users based on certain resource usage rules in a specific resource environment based on cloud computing analysis. In this article, a framework of cloud and fog hybrid network for Community Internet of Things is proposed, which solves the problem of high latency of data processing in the cloud [17]. In the actual production range, routers, switchboards, and other peripheral devices are used to create a layer of fog between the cloud server and manufacturing equipment. In order to solve the problem of insufficient computing power of the optical gyroscope node, a multi-functional distributed computing method and an algorithm based on the simulated annealing algorithm to balance the load of the particle swarm are proposed to achieve the goal of minimum task processing delay [18].

Regarding the multi-cluster edge cloud, two technical points need to be paid attention to: one is resource allocation, and the other is load balancing. Therefore, when multi-cluster edge cloud is applied to communities, two points need to be considered: first, reasonable allocation of outdoor resources in communities; second, load limitation of outdoor facilities in communities. This article will separately introduce planning strategies that consider time characteristics and that do not consider time characteristics in a multi-cluster edge cloud, so as to effectively allocate resources and solve the problem of balancing load. One characteristic of delay-sensitive applications is that it must respond to user needs within a specified time. In order to achieve this goal, this paper adopts the gray model and weighted model dynamic scaling strategy, and finally summarizes an active dynamic scaling strategy GMHPA. Based on the analysis of the health data of the actual monitoring community residents, a reasonable prediction model was selected according to the trend of the data, and the sample data were obtained, so as to improve the service quality of the community cloud resource mechanism and ensure the balanced operation of the cloud resource scheduling mechanism in the community space. Combined with the big data of community residents' health, this scheduling mechanism can fully deploy community resources, so that residents can make use of community resources to save themselves in time when health problems occur. For each request, peripheral applications must occupy a certain amount of system resources for processing, which is the computing power that the application obtains from the edge cloud through virtualization technology. The community cloud scheduling mechanism, combined with residents' health data and community Internet of Things, is conducive to guiding the rational allocation of community resources, creating health-promoting community outdoor space, and helping residents to timely use community resources to save themselves when health problems occur. For each request, the peripheral application must consume a certain amount of system resources to process, which is the computing power that the application obtains from the edge cloud through virtualization technology, as shown in formula (1):

(1) $$\begin{array}{c} t_{2}=\frac{\text{ size}}{{\text{mips}}_{v}}. \end{array}$$

Since vertical scaling changes the size of the resource quota of the application, the resource quota of the application may be too large, and the general resources of the physical node may be insufficient. Especially in the edge environment, the limited resources of the node make it impossible for the node to complete the resource allocation. In addition, vertical expansion usually requires restarting the application, which may cause service interruption. Therefore, we should focus on the service coverage of the edge of community outdoor space, and strictly prevent the problems of insufficient resource allocation and low security of community outlying space. This article uses the horizontal scaling method to solve the problem of resource planning in delay-sensitive attachments. In the horizontal scale, the overall computing power of the application is proportional to the number of copies of the application. Since the total resources of each peripheral group are limited, the requirements of the current application program need to be completed in different time periods to achieve the actual number of resources required by the application program, as shown in formula (2):

(2) $$\begin{array}{c} \text{mips}=n\times {\text{mips}}_{v}. \end{array}$$

The set of three applications is shown in formula (3):

(3) $$\begin{array}{c} \begin{array}{c} A^{s}=\left\{A_{1}^{s},A_{2}^{s},\ldots ,A_{N}^{s}\right\}\\ A^{u}=\left\{A_{1}^{u},A_{2}^{u},\ldots ,A_{M}^{u}\right\}\\ \;A^{p}=\left\{A_{F_{1}}^{p},A_{F_{2}}^{p},\ldots ,A_{F_{K}}^{p}\right\} \end{array}. \end{array}$$

For latency-sensitive applications, only move within the cluster, not between groups. Therefore, the same application in different groups can be regarded as irrelevant, and Definition 2 does not lose its general meaning. For any delay-sensitive application, suppose the number of copies is *k*, as shown in formula (4):

(4) $$\begin{array}{c} A_{n}^{s}=\left\{c_{n.1},c_{n,2},\cdots \cdots ,c_{n,K}\right\}. \end{array}$$

Only consider the CPU and RAM that have the greatest relationship with the calculation and the resource dimension, as shown in formula (5):

(5) $$\begin{array}{c} D=\left(\text{cpu},\text{ram}\right). \end{array}$$

The resources that a single node can provide are shown in formula (6):

(6) $$\begin{array}{c} C_{f_{i,j}}^{D}=\left(C_{f_{i,j}}^{\text{cpu}},C_{f_{i,j}}^{\text{ram}}\right). \end{array}$$

For delay-insensitive applications, as shown in formula (7):

(7) $$\begin{array}{c} \rho_{A_{m}^{\prime \prime }}^{C}+\underset{i\in l}{\sum }\underset{j\in J}{\sum }\rho_{A_{m}^{\prime }}^{f_{i,j}}=1. \end{array}$$

Calculate the utilization rate of application resources by the following formula (8):

(8) $$\begin{array}{c} \text{cur Metric Value}=\frac{\sum_{i}^{n}\text{metric }{\text{Value}}_{i}}{n\times \text{request Value}}. \end{array}$$

Formula (8) is used to calculate the utilization rate of outdoor facilities in the community, and the frequency of use of various spaces in the community is studied to provide basic data for future resource allocation.

Use the following formula (9) to calculate the expected number.

(9) $$\begin{array}{c} \text{Replicas}=\text{ceil}\left[\text{cur Replicas}\times \left(\frac{\text{cur Metric Value}}{\text{desired Metric Value}}\right)\right]. \end{array}$$

Compare the resource expectation obtained in formula (9) with the actual resource distribution to find out the data difference, and take the difference value as the basis for guiding the community resource allocation.

The *n* sampling values taken out periodically are recorded as formula (10):

(10) $$\begin{array}{c} x^{\left(0\right)}=\left[x^{\left(0\right)}\left(1\right),x^{\left(0\right)}\left(2\right),\cdots ,x^{\left(0\right)}\left(n\right)\right]. \end{array}$$

The order ratios of the sampling sequence are calculated by formulas (11) and (12). If all the order ratios of the sequence fall within the interval, the gray model can be used to model and perform translation conversion.

(11) $$\begin{array}{c} \lambda \left(k\right)=\frac{x^{\left(0\right)}\left(k-1\right)}{x^{\left(0\right)}\left(k\right)} \end{array}$$

(12) $$\begin{array}{c} x^{\left(0\right)}\left(k\right)=x^{\left(0\right)}\left(k\right)+c,k=1,2,\ldots ,n. \end{array}$$

Carry out a cumulative sum, as in formula (13):

(13) $$\begin{array}{c} x^{\left(1\right)}=\left[x^{\left(1\right)}\left(1\right),x^{\left(1\right)}\left(2\right),\cdots \cdots ,x^{\left(1\right)}\left(n\right)\right]. \end{array}$$

Use the first-order accumulation sequence to establish a differential formula through formula (14):

(14) $$\begin{array}{c} \frac{dx^{\left(1\right)}}{dt}+ax^{\left(1\right)}=b. \end{array}$$

Then, use formulas (15) and (16) to solve the parameters.

(15) $$\begin{array}{c} B=\left[\begin{array}{cc} -\frac{1}{2}\left[x^{\left(1\right)}\left(2\right)+x^{\left(1\right)}\left(1\right)\right] & 1\\ -\frac{1}{2}\left[x^{\left(1\right)}\left(3\right)+x^{\left(1\right)}\left(2\right)\right] & 1\\ \ldots & \ldots \\ -\frac{1}{2}\left[x^{\left(1\right)}\left(n\right)+x^{\left(1\right)}\left(n-1\right)\right] & 1 \end{array}\right], \end{array}$$

(16) $$\begin{array}{c} \hat{u}=\left[\begin{array}{c} a\\ b \end{array}\right]={\left(B^{T}B\right)}^{-1}B^{T}Y. \end{array}$$

By solving the first-order ordinary differential formula, formula (17) can be obtained:

(17) $$\begin{array}{c} x^{\left(1\right)}\left(k+1\right)=\left[x^{\left(0\right)}\left(1\right)-\frac{b}{a}\right]\times e^{-ak}+\frac{b}{a},k=1,2,\ldots \ldots ,n. \end{array}$$

The predicted value can be restored as formula (18):

(18) $$\begin{array}{c} x^{\left(0\right)}\left(k+1\right)=x^{\left(1\right)}\left(k+1\right)-x^{\left(1\right)}\left(k\right)=\left(1-e^{a}\right)\left(x^{\left(0\right)}\left(1\right)-\frac{b}{a}\right)e^{-ak},k=1,2,\cdots ,n. \end{array}$$

The weighted moving average prediction model directly uses formula (19) to calculate the predicted value at the next moment. It can be seen that the weighted moving average model can effectively reflect the recent average value of the time series sequence.

(19) $$\begin{array}{c} x^{\left(0\right)}\left(k+1\right)=\beta_{1}x^{\left(0\right)}\left(1\right)+\beta_{2}x^{\left(0\right)}\left(2\right)+\cdots +\beta_{k}x^{\left(0\right)}\left(k\right),\beta_{1}+\beta_{2}+\cdots \beta_{k}=1. \end{array}$$

The GMHPA strategy establishes a load queue for the application as historical data, and uses the gray model in each monitoring cycle to predict the load usage of the application in the next cycle. According to the comparison between the forecast result and the collection result of this cycle, when the forecast amount is greater than the current acquisition amount, the load is considered to have an upward trend, and the forecast amount is used as the input of the HPA strategy. In addition, when the predicted amount is less than the current collected amount for many consecutive times, the load is considered to have a downward trend, and the predicted amount is used as the input of the HPA strategy. Otherwise, the historical data are predicted by moving weighted average and this result is selected as the input of the HPA strategy. Obviously, when the queue length of the moving weighted average model is 1, the GMHPA strategy degenerates into the same responsive shrinkage as the HPA strategy when shrinking.

The amount of S resources in the cluster can be calculated by the formula (20):

(20) $$\begin{array}{c} C_{F_{i}}^{D}=\underset{j\in J}{\sum }C_{f_{i}}^{D}=\left(\underset{j\in J}{\sum }C_{f_{i}}^{\text{cpu}},\underset{j\in J}{\sum }C_{f_{i}}^{\text{ram}}\right). \end{array}$$

The amount of used resources in the cluster is as shown in formula (21):

(21) $$\begin{array}{c} R_{F_{i}}^{D}=\underset{n\in N}{\sum }R_{A_{n}^{s}}^{D}+\underset{m\in M}{\sum }R_{A_{m}^{\prime \prime }}^{D}+R_{A_{i}^{\prime }}^{D}=\underset{n\in N}{\sum }\underset{k\in K}{\sum }R_{c_{n,k}}^{D}+\underset{m\in M}{\sum }\rho_{A_{m}^{\prime \prime }}^{F_{i}}R_{A_{m}^{\prime \prime }}^{D}+R_{s_{r}^{r}}^{D}. \end{array}$$

At this time, there are formulas (22) and (23):

(22) $$\begin{array}{c} R_{F_{i}}^{\text{cpu}}=\underset{n\in N}{\sum }\underset{k\in K}{\sum }R_{c_{n,k}}^{\text{cpu}}+\underset{m\in M}{\sum }\rho_{A_{m}^{u}}^{F_{i}}R_{A_{ni}^{u}}^{cpu}+R_{A_{F_{i}}^{pu}}^{\text{cpu}}, \end{array}$$

(23) $$\begin{array}{c} R_{F_{i}}^{\text{ram}}=\underset{n\in N}{\sum }\underset{k\in K}{\sum }R_{c_{nk}}^{\text{ram}}+\underset{m\in M}{\sum }\rho_{A_{m}^{j}}^{F_{i}}R_{A_{m}^{\prime \prime }}^{\text{ram}}+R_{A_{F_{i}}^{p}}^{\text{ram}}. \end{array}$$

The resource utilization rate of cluster *i* can be calculated from the total resource amount and the used resource amount as shown in formula (24):

(24) $$\begin{array}{c} \theta_{F_{i}}^{D}=\frac{U_{F_{i}}^{D}}{C_{F_{i}}^{D}}=\frac{C_{F_{i}}^{D}-R_{F_{i}}^{D}}{C_{F_{i}}^{D}},0<\theta_{F_{i}}^{D}<1. \end{array}$$

At this time, it is as formula (25):

(25) $$\begin{array}{c} \theta_{F_{i}}^{\text{cpu}}=\frac{U_{F_{i}}^{\text{cpu}}}{C_{F_{1}}^{cpu}}=\frac{C_{F_{i}}^{cpu}-R_{F_{i}}^{\text{cpu}}}{C_{F_{i}}^{\text{cpu}}},0<\theta_{F_{i}}^{cpu}<1. \end{array}$$

According to the data obtained by formula (25), allocate resources reasonably for each space in the community, improve the layout of community resources, and finally maximize the utilization rate of community outdoor resources.

In this paper, air pollution parameters, air concentration parameters, air humidity parameters, water quality parameters, community sound parameters, community light parameters, community temperature parameters, community health parameters, community service facilities parameters, and community fitness space parameters are used as basic data. Through the above calculation process in different areas, it is concluded that the community of air purification facilities allocation rate, water environment purification system deployment rate, noise reduction space allocation rate, shading space allocation rate, heating facilities allocation rate, barrier-free space allocation rate, outdoor fitness space allocation rate, walking outdoors space allocation rate, and outdoor landscape utilization rate of community public resource allocation. According to the final calculation results, this paper detects whether the environmental quality of the community is healthy, and allocates the outdoor resources of the community reasonably. The real-time management of community resources rationalizes the distribution of community outdoor resources, and finally builds a sustainable development of health promotion community.

### 2.2. Community Internet of Things Technology

Community Internet of Things Technology is the community system of things and things, which connects the community material information with the Internet through information sensing equipment, and constructs the community Intranet for information exchange, so as to realize the intelligent identification and management of the community. Apply community IoT technology to the construction of community outdoor space, which can feed back the frequency of outdoor facilities' use and community health parameters of community members in real time and upload this information to the community cloud system in real time. Through these measures, we can observe the dynamic trend of community outdoor space and make the community resource allocation mechanism more reasonable. The application of Internet of Things technology can effectively optimize the outdoor physical space environment of the community, improve the vitality of the outdoor space, and form a healthy community physical space environment, which is conducive to guiding the community residents to get out of the indoors, carry out communication, and indulge in sports, leisure, and entertainment, so as to promote the physical and mental health of the community residents and form a healthy community atmosphere.

Intelligent community will be the overall trend in future community planning. For the intelligent Community Internet of Things technology, its specific manifestations are twofold. First of all, sensors or other sensing terminals used in the underlying data collection and perception layer of the Community Internet of Things should gradually develop towards miniaturization and intelligence, which can lay a solid and intelligent foundation for the Community Internet of Things technology. Secondly, for the control system, while ensuring the safety of the system platform, its shareability should be gradually improved, so as to facilitate the perception of the health status of family members and realize the rescue across the space.

The SAPSO-LB algorithm based on ITCFN needs to set initial condition parameters in the simulation test operation, and the setting of the parameters fully meets the reliability, logic, and scientificity; this feature is beneficial to obtain more accurate community material information and to analyze the health needs of community residents, so that the proposed scheme can be found in a limited number of iterations for the optimal solution. The specific process is shown in Table 1. The basic parameters of the algorithm are set as follows: the number of groups N is 200, the learning factor C1 is 2.0001, the learning factor C2 is 2.2001, the annealing constant inertia weight LAMDA is 1, the maximum number of iterations *M* is 1000, and the search space dimension *D* is 10.

In order to verify the effectiveness of the proposed algorithm, the data processing time delay is compared with traditional cloud computing and a single fog computing node. The task amount is set to 0-20 GB. Simulation comparison is performed based on the built model to solve the same task.

In order to study the influence of the number of fog nodes in the fog computing layer on the data processing delay, when the total amount of data *X* is 4 Gb, 8 Gb, 12 Gb, 16 Gb, and 20 Gb, the number of fog computing nodes is 1–10. Through simulation experiments, the results of the delay required for processing data with different numbers of nodes are solved.

In order to study the effectiveness of the data delay algorithm, the SAPSO-LB algorithm is compared with classic load balancing algorithms such as the MPSO-CO algorithm, weighted round-robin method, Pick-KX algorithm, and greedy load balancing algorithm. The selected data volume is 0- 20 GB; through simulation experiments, the results of the processing delay required by different algorithms to process the same amount of data are solved.

Through the above algorithm, the data information of outdoor material space in each community is obtained. The collected spatial information mainly includes community air quality information, community water body information, community sound information, community lighting information, community temperature information, community accessibility facilities use information, fitness space use information, community outdoor recreation facilities use information, community health information, etc. Eventually, this information will be uploaded to the community cloud system to form the initial community environmental detection results.

In this paper, the service area of community Internet of Things is the outdoor space in the community, and the main service object is community residents. The main purposes of establishing the community Internet of Things include the following three points: firstly, to test the health degree of the community environment preliminarily; secondly, to collect information and pass to the community cloud scheduling mechanism; the third point is to lay a solid foundation for the rationalization of subsequent community resource scheduling.

## 3. Community Environment Detection Based on Cloud Resource Scheduling Mechanism

### 3.1. Analysis of the Livability of the Environment Outside the Community

The environment outside the community mainly includes material space and human environment. The main reference data of cloud resource scheduling mechanism of community outdoor space include six elements: air quality parameters, water environment parameters, community comfort, fitness space utilization rate, community service facility utilization rate, and community residents' health parameters. The main reference data of cloud resource scheduling mechanism of community outdoor space include five elements: air quality parameters, water environment parameters, community comfort, fitness space utilization rate, and community service facility utilization rate. Among them, the combination of Internet of Things technology and cloud computing is extremely important. The original computing information of air quality, water environment, community comfort, fitness space utilization rate, community service facility utilization rate, and community health parameters mainly comes from the information collection of community intelligent devices. Among them, air quality includes pollution source, concentration limit, and monitoring three criteria layer; water environment includes three criteria layers: water quality, water body, and water safety. Community comfort level includes sound, light, heat, suitable for the old and suitable for the young. Fitness space utilization rate includes three standard levels: gymnasium, outdoor fitness space, and outdoor amusement ground. Utilization rate of community service facilities mainly includes management, frequency of use, and allocation.

Through intelligent community information collection, the community material space information is transmitted to the community cloud system. After data processing, the distribution of community resources can be found. Through the community cloud resource scheduling mechanism, resources can be deployed in time to meet the health needs of community residents. The interaction between community intelligent IOT and cloud scheduling mechanism can monitor community environmental quality in real time, so as to effectively maintain a health-promoting community environment in the long term.

### 3.2. Community Livability Monitoring Model Construction

The literature proposes a multi-layer cloud boundary management system based on the principle of obedience. Its framework is mainly divided into two parts: cloud cluster and collaboration layer [19]. The former undertakes a certain amount of work, while the latter is responsible for managing marginal groups and peripheral applications. In this system, peripheral applications are divided into two categories: delay-sensitive and delay-insensitive [20]. Requests for delay-sensitive applications are directly processed in the cloud layer near the boundary, while requests for delay-sensitive applications are effectively processed through the communication layer, which ultimately solves the application positioning problem under multi-cluster edge cloud collaborative scheduling. In the framework of this program, the literature studies the problem of planning resources for time-sensitive applications [21]. Since delay-sensitive applications usually require high-quality services, the dynamic expansion strategy to cope with pressure changes has a lag in peripheral conditions and cannot provide effective service guarantee. Therefore, based on the gray model and the weighted model dynamic scaling strategy, this paper proposes an active dynamic scaling strategy GMHPA, which uses the gray model to predict workload and determines the trend of load changes based on actual monitoring indicators. Then, according to the changing trend, different prediction models will be selected to calculate the number of samples.

In addition, the experimental results show that, compared with the current response strategy, GMHPA's increased workload strategy can effectively expand the capacity of time-sensitive applications in advance, and reduce the workload, so as to better meet the quality of service requirements. In order to improve the overall efficiency of the use of cluster resources, the literature has developed a resource management strategy for different cluster groups. The strategy is divided into three stages: one is to classify according to the degree of load usage; the second is to classify according to the results, and the scheduling application is selected according to the control trigger of the load group; and the third is to assign a target group to the application planner. The experiment shows that the DICCS strategy can effectively execute the function of inter-cluster planning to adapt to insensitive time applications, improve the efficiency of cluster resources, and ensure load balance between groups. The literature introduces information search technology, such as data analysis, metadata extraction, and format conversion. The storage method is mainly based on the data type and the corresponding characteristics of the data to select the corresponding storage location. Different types of systems need to store and divide data operations such as selection and search. The literature proposes intelligent terminals. For intelligent industrial Internet of Things technology, its specific manifestations are in two aspects. First of all, sensors or other sensing terminals used in the underlying data collection and perception layer of the Industrial Internet of Things should gradually develop towards miniaturization and intelligence, which can lay a solid and intelligent foundation for the Industrial Internet of Things technology. Secondly, for the control system, its shareability is gradually increased while ensuring the safety of the system platform, so that other systems can cross-platform mutual assistance with the control system.

The system basically covers all aspects of natural, humanistic, and social factors in the evaluation index system of outdoor space in cold region communities, and they also coordinate and interact with each other.

## 4. Health Promotion in Community Outdoor Space Planning

### 4.1. The Impact of Community Outdoor Space Health

With the continuous improvement of national living standards in recent years, people's needs for spiritual life are gradually increasing. At the same time, in the process of rapid urbanization and rapid changes in urban communities, the impact of residents' spiritual life is also very huge. At present, the community psychology and community network of residents in the residential environment need to be reconstructed. The mental loneliness, indifference, depression, and other problems of urban residents need to be alleviated or even eliminated through the joint efforts of urban communities and residential community environment construction. As the current domestic development and renovation of residential areas pay more attention to the environmental quality of physical space, but relatively neglect the environmental quality of the community and its construction, this has caused the unbalanced development of the two. Therefore, it is necessary to have more understanding, knowledge, and research on the relevant elements of building a healthy residential community environment. The expansion elements of community environmental health based on community networks, including loneliness, belonging, participation, and pride, are closely related to community networks in population areas. Therefore, it must be guided by the cultural factors of its residential community. Yuan Yuan pointed out that unity is the ultimate determinant of environmental stability and balanced development, and it is also the ultimate criterion for measuring residents' evaluation of the community's environment. Under the market situation, the settlement that a resident finally chooses should be based on a combination of multiple factors, and the chosen place of residence that best meets his or her needs and is the most satisfactory.

Relevant experts believe that if the relevant environmental factors of the residential area are combined with the residents' psychological assessment, an external spatial environment can be established accordingly, and it can be matched with the psychological needs of the residents. Only when residents mentally evaluate their health can they ensure that the community's living environment is in a healthy and functioning state. This article believes that the basic elements and expansion elements of community structure content are very important to the environmental impact of residential communities. Although they have their own focuses, the construction of these two types of elements also promotes and influences each other. The construction and operation of each type of element will have an impact on the construction of other elements. Only when the design needs of various environmental factors are correspondingly met can the environmental quality of the community be fundamentally improved and the good neighborly relationship between residents be promoted. In fact, for the construction of community environmental health, we must find a solution from the material space level, so that it will not become a “paper talk,” and the residents' various needs for the community environment construction in the residential area can be implemented. Fundamentally improve the outdoor space environment of residential areas and the quality of community environment. Therefore, the design and research of the outdoor space environment of residential areas under the value orientation that meets the requirements of the construction of the above-mentioned community environmental health impact elements is to solve the content of how to design and set up the physical space environment, so as to promote the formation of a healthy and good community environment, and to build a healthy and harmonious organic unity of outdoor space environment and community environment in residential areas. According to the survey of the most satisfied and dissatisfied contents in the community, it can be found out which residential and environmental issues the residents are most concerned about, and the important influencing factors can be summarized by analyzing these issues. The results are summarized in Table 2.

The “most sensitive and important content” in Table 3 are the most urgent and important issues or services at the moment. They are the priority elements and should be met during the residential area construction phase. Many of these issues are mainly related to the physical space of the residential area. However, it must be pointed out that this is also closely related to the scope of the community's environmental impact. What is important is that “safe environment” corresponds to the “personal” element of “property management,” and “community interaction” corresponds to the “participation” element. Therefore, a preliminary conclusion can be drawn: First, the residents are very concerned about public facilities, environmental quality, parking lots, public health and other issues, which shows that the current residents' requirements for the community living environment remain high. Second, residents also attach great importance to housing management, property management, community relations, and other issues, which mean that after meeting material needs to a certain extent, people will inevitably begin to deal with the nonmaterial aspects of spiritual needs. Then, people will care for the specific issues related to the community environment and other health impact factors mentioned in this article, as shown in Table 3.

According to statistics, the population is mainly composed of young and middle-aged people. It should also be pointed out that according to the relevant internationally recognized standards, the community is now in an aging situation. It can be seen from Table 4 that the occupation of the population is diversified.

The survey shows that the proportion of families without children in the community is relatively high, and some families are older married couples. As shown in Table 5, it can be seen that the proportion of households with three members is the highest, and the proportion of households with more than four is the lowest.

### 4.2. Community Outdoor Space Planning and Design Based on Health Promotion

#### 4.2.1. Design Guidelines

Health is the eternal theme of mankind. The World Health Organization defines health as “not only to get rid of disease and weakness, but also to maintain a normal state of physical, mental and social development.” Whether in China or Western countries, people desire health and comfort. The Warsaw Declaration called for construction to enter the era of environmental protection. Over the past 20 years, overseas housing development has been divided into three stages: energy conservation, environmental protection, and comfort and health. Countries have adopted energy conservation initiatives, and people have gradually realized that the Earth's environment is closely related to the survival of mankind. The basic conditions of human life are comfort and health, to achieve a healthy and comfortable life, and it is inseparable from the following six categories: basic environmental infrastructure, green landscape, activity locations, roads, vehicle parking, and public facilities, each of which continues to be subdivided into several subcategories.

(1) Basic environmental facilities: Environmental infrastructure is an important measure to improve the outer space environment and the landscape quality of residential areas. It develops rapidly through small investment, rapid return, small area, and high flexibility. Such facilities need to be reasonably configured in various types of places in outdoor spaces. It plays an important role in improving people's interest in life and quality of life, shaping a favorable outdoor environment image, and promoting communication between neighbors.

(2) Greening landscape: Greening landscape includes two aspects: planting and green space. Planting refers to the selection of plant species, mainly for the selection of tree species; turf; flower size, shape, color, height, and other characteristics. Plants can be used as an auxiliary to the formation of outer space. Green landscape can be used for public buildings, and green land is part of the public building complex. The green road is basically a landscape function, and the green house is a landscape and ecological function. These regulations are particularly applicable to the guiding principles of public green zone planning, including in parks, small gardens, green zone groups, and green areas near houses.

(3) Event venue: The activity venues involved in this article mainly adopt hard pavement to provide residents with outdoor activity space and necessary entertainment facilities. This is the main place for residents to perform leisure activities, the focus of the construction of community livability, and also the key area of the model structure. Through the scientific layout of the event venues, the utilization efficiency of the event venues can be better improved and the optimal allocation of space can be realized.

(4) Community cloud resource scheduling mechanism and the application of community IoT technology: This article mainly involves the cloud and fog hybrid network framework and intelligent Internet of Things technology to realize real-time feedback of community information. More importantly, they can monitor the health promotion effects of space planning in real time. Through the establishment of the monitoring system through the Internet of Things, service personnel can discover various potential risks in the first time, and grasp the changes in the community environment, so as to choose the most optimized service plan.

#### 4.2.2. The Goal of the Overall Design

(1) System construction and evaluation: Establish an evaluation system that combines the community cloud dispatch mechanism with the community Internet of Things, monitor the status quo of the community environment in real time, deploy community materials in real time, rationally allocate community outdoor facilities, guide community residents to exercise, communicate, and relax outdoors, and create a health-promoting community outdoor space environment.

Apply community Internet of Things technology, barrier-free facilities, children's outdoor activity space, fitness space, and other places to reasonably arrange health data sensing devices, detect abnormal health data of community residents, identify sudden health problems of community members, and upload physical data to geographic locations. The community cloud system facilitates the dispatch of emergency resources.

Based on the above research on the cloud resource scheduling mechanism and the Internet of Things, the health effects of the cloud resource scheduling mechanism and the Internet of Things in the community outdoor space planning are discussed. Remote health monitoring system based on community Internet of Things technology is used to achieve rapid rescue across spaces, monitor the health data of community residents in real time, explore the influence factors of community outdoor space on health, and guide space planning.

(2) Key issues in design: In order to ensure the high-quality materials required for the building space environment, from the external environment function to the outer space design to the landscape design, higher fire protection standards must be met. In addition to meeting basic physiological needs (solar energy, ventilation, day-lighting, etc.), transportation and external environmental facilities, as well as the needs of vulnerable groups such as the elderly, children, and the disabled should also be considered. The outdoor space environment should be considered.

Create a good shape and image, improve the external space of the house in an aesthetic physical environment, and provide high-quality materials for the building space environment. From the external environment function to the outer space design and landscape design, the goal must be a higher standard. In addition to meeting the basic physiological standards such as sunlight, ventilation, lighting, and fire prevention, other basic standards such as building quality should also be considered. The behavior of people, traffic environment, and outdoor furniture design for different groups of people should be considered. One of the main design goals is to create the environment. The most direct requirement of spatial form is people's demands for spatial function and aesthetics to meet the basic requirements of the architectural space environment of residential areas.

(3) Development trends in design: The foundation of a healthy life is human health. Health includes not only physical health in daily life but also mental health. It is necessary to promote healthy diet of residents, strengthen physical exercise, build various sports venues, and promote the improvement of residents' health. Mental health encourages a positive attitude towards life and values. A diversified communication space should be created, with cultural background and humanistic spirit, to promote connection, safety, and pride between communities. By creating an outer space environment in the residential area, the life of the residents is guaranteed from the material and space perspective.

In today's era, people mostly pursue higher-level designs and are very concerned about the health of the community environment. Therefore, we should attach importance to environmental protection, advocate a healthy lifestyle, and provide people with medical services and a good health environment in the community. This can make people feel safe and feel that they are part of the community, so that residents have a good sense of security, identity, and belonging in their lives. It can also regularly assess the psychological status of community residents, maintain a healthy and harmonious lifestyle in the society, make people feel proud of the overall evaluation of the community, and generate a desire for permanent residence.

## 5. Conclusion

This article analyzes the related issues brought about by China's rapid urbanization and social transformation, conducts extensive social research on the relationship between influencing factors, and explores community outdoor space and environment testing. This article integrates the cloud resource control mechanism and the Internet of Things into the community outdoor space planning to effectively improve the rate of health promotion in community construction. In this article, according to the actual needs of the site and the architecture of the industrial Internet of Things technology, a remote monitoring project for outdoor large-scale equipment carts is developed, a corresponding solution is developed, and a remote monitoring system is developed for the industrial Internet of Things technology. The software and hardware platforms of the system have been tested on-site, and on-site data can be displayed remotely. After the data are uploaded to the community cloud, the cloud scheduling mechanism reasonably schedules outdoor resources based on the data to meet the life needs of community members. After planning the outdoor space in the community according to the above strategy, good social communication conditions have been created, related community communication issues have been effectively managed, communication between residents has been promoted, and a social atmosphere of mutual assistance and love among neighbors has been created in the traditional sense.

Based on this, this article introduces the relevant spatial factors that affect the health of social members, and through relevant calculation and analysis, on the basis of constructing the factors that affect the health of the community, it discusses the design standards of outdoor space environment based on cloud resources. Scheduling mechanism. It is hoped that on the basis of the basic element structure requirements of the community area, the construction of elements related to the social environment and health will be improved, and the design requirements of these elements will be used as guidance. The outer space design guarantees residents' physical, psychological, and spiritual health needs at multiple levels. In this way, we will promote the sustainable development of China's human settlement environment, further improve and enhance the quality of human settlements, and create a comfortable and healthy human settlement environment. The whole system provides a solid theoretical foundation and useful technical exploration for the remote monitoring of large outdoor equipment. The innovative points of this plan are: Firstly, to promote the intelligent process of community environment detection, and regularly check the health of the community's outdoor space; secondly, it is to set up reasonable health data sensing equipment for community members, so that residents can save themselves; thirdly, real-time deployment of community outdoor resources is meant to meet the health needs of community members, and create a health-promoting community outdoor space environment.

## Figures and Tables

**Table 1:** Fog node equipment parameters.

Parameter	Z1	Z2	Z3	Z4	Z5	Z6	Z7	Z8	Z9	Z10
*λ*_zi_	2	1	3	0.5	0.4	0.5	0.7	0.3	0.5	1
*τ*_zi,zj_	0	0.11	0.08	0.13	0.07	0.08	0.05	0.05	0.12	0.13

**Table 2:** “What are the three things you are most satisfied with in the community?”

Sensitivity number	Project description	Number of answers (parts)	Importance score (points)
1	Responsible for security work	48	100.0
2	Good environment	45	93.7
3	Health	35	73.4
4	Better greening	28	59.4
5	Good property management	22	44.8
6	Fitness facilities	10	20.1
7	Beautiful landscape	9	18.8
8	Other	8	15.3

**Table 3:** List of the most concerned issues of community residents.

Serial number	The most sensitive and important content
1	Safe atmosphere
2	Public facilities service
3	Parking problem
4	Environmental sanitation
5	Green landscape
6	Fitness facilities
7	Property management
8	Noise problem
9	Community activities, contacts
10	Housing quality

**Table 4:** Occupational composition of residents in the community.

Occupation category	Constitute percentage	Occupation category	Constitute percentage
Party and government officials	4	Self-employed persons	17
Business management personnel	7	Industrial transportation	4
Managers of institutions	5	Business services	13
Company owner/shareholder	8	Military police	1
Scientific research and technical personnel	5	Student	2
Arts and sports workers	0	Agricultural production	0
Lawyer	0	Retired/retirees	4
Medical workers	4	Housewife	4
Educators	8	Laid-off/unemployed	2
Press and publication staff	0	Migrant workers	2
No fixed/freelancer	5	Other	3
Total		100%	

**Table 5:** Resident population of households in the community.

Permanent household population	Percentage
1 person	2
2 people	24
3 people	55
4 people	12
4 people or more	7
Total	100

## Data Availability

The datasets used and/or analyzed during the current study are available from the corresponding author on reasonable request.
